The article "A structured review of reasons for ecstasy use and related behaviours: pointers for future research" was published in 2009. Journal: BMC Public Health.

# A structured review of reasons for ecstasy use and related behaviours: pointers for future research

**DOI:** 10.1186/1471-2458-9-230

**Published:** 2009-07-13

**Authors:** Gjalt-Jorn Ygram Peters, Gerjo Kok

**Affiliations:** 1 Department of Work and Social Psychology, Faculty of Psychology and Neuroscience, Maastricht University, Maastricht, The Netherlands

## Abstract

**Background:**

While the health risks of using ecstasy warrant intervention development, a recent meta-analysis of determinants of ecstasy use identified a number of lacunae in the literature. Specifically, no studies were included that address behaviours other than 'using ecstasy' (e.g. 'trying out ecstasy' or 'ceasing ecstasy use'). However, because meta-analyses aim to integrate study results quantitatively, the resulting rigid exclusion criteria cause many studies to be discarded on the basis of their qualitative methodology. Such qualitative studies may nonetheless provide valuable insights to guide future research. To provide an overview of these insights regarding ecstasy use, the current study summarizes and combines what is known from qualitative and exploratory quantitative literature on ecstasy use.

**Methods:**

The databases PsycINFO and MedLine were searched for publications reporting reasons for ecstasy use and related behaviour, and the results were structured and discussed per behaviour and compared over behaviours.

**Results:**

Two main categories of reasons were found. The first category comprised reasons to start using ecstasy, use ecstasy, use ecstasy more often, and refrain from ceasing ecstasy use. The second category comprised reasons to refrain from starting to use ecstasy, use less ecstasy, and cease using ecstasy. Reasons for related behaviours within each of these two categories appear to differ, but not as substantially as between the two categories. A large number of reasons that were not yet explored in quantitative research emerged.

**Conclusion:**

The current summary and combination of exploratory studies yields useful lists of reasons for each behaviour. Before these lists can inform interventions, however, they beg quantitative verification. Also, similarity of determinant configurations of different behaviours can be assessed by addressing determinants of several behaviours in one study. Another important finding is that meta-analytical integration of the literature may overlook important findings and implications. Thus, qualitative reviews remain useful instruments in setting the research agenda.

## Background

Although evidence that ecstasy use may be damaging to health accumulates [1,2], its prevalence persists [3,4]. Theory-based behavioural interventions have successfully generated behaviour change in other areas [5,6], and may likewise have beneficial effects when applied to ecstasy use. However, development of an effective intervention requires knowledge about which modifiable determinants need to be targeted [7]. A recent meta-analysis of quantitative studies on ecstasy use and related behaviours, which aimed to provide this knowledge, concluded that much research is still necessary [8]. Specifically, of all behaviours relevant to ecstasy use (e.g. trying out ecstasy, applying harm reduction strategies, ceasing ecstasy use) only the broad behavioural category of 'using ecstasy' had been addressed by the included studies. Because meta-analyses aim to quantitatively integrate the literature, they generally exclude studies that do not report certain statistics. For example, the meta-analysis about ecstasy use included only studies that "assess quantitatively the relationship between determinants and behaviour or intention" [[8], p. 110]. These restrictive inclusion criteria led to the exclusion of all qualitative and exploratory studies into the reasons for ecstasy use, while paradoxically, it is exactly this exploratory methodology that renders these studies particularly valuable in setting the research agenda. The current review sets out to inform future research into ecstasy use and related behaviours by summarising this qualitative and exploratory quantitative literature.

Although the aforementioned meta-analysis did result in a list of determinants that seem relevant for ecstasy use (i.e. attitude, subjective norm, perceived behavioural control, moral norm, anticipated regret and habit), consideration of the most salient underlying beliefs indicated that some of these determinants of ecstasy use may prove exceptionally hard to modify [8]. For example, although ecstasy users had a higher descriptive norm than non-users (i.e. users perceived there to be more ecstasy use at dance events), this difference appeared to reflect an *under*-estimation of actual ecstasy use prevalence on the part of non-users. In this case, therefore, correcting this erroneous belief would lead to *more *ecstasy use, and an intervention aiming to decrease descriptive norms among ecstasy users would have to present incorrect information about the prevalence of ecstasy use (i.e. portray ecstasy use prevalence as lower than it is). The difficulties of intervening on the reported determinants seem to be underlined by a recent evaluation of an intervention among ecstasy users, where the authors concluded that a brief motivational intervention was no more efficient than the information-only control condition [though use decreased in both conditions, which most control participants attributed to the self-assessment at baseline; [9]]. In addition, none of the reviewed studies specifically addressed the initiation or cessation of ecstasy use or the application of harm reduction strategies. All studies addressed the broad behavioural category of 'using ecstasy' [e.g. by comparing users with non-users, or examining the intention to 'use ecstasy'; [8]], which may be problematic because determinants of related but different behaviours such as these are assumed to differ [7,10]. Finally, it seemed that the summarized research had not addressed a number of potentially relevant determinants [8].

Thus, so far, only one of several relevant behaviours has been reviewed; the identified determinants appear hard to modify; and relevant determinants may have been omitted. The current paper investigates whether studies into other ecstasy use-related behaviours or addressing other determinants do exist, but were excluded by the rigid exclusion criteria of the meta-analysis drawing these conclusions. Specifically, the current paper reports a structured review of all qualitative studies and exploratory studies, which did not report an association with intention or behaviour but did report reasons for performing (or not performing) an ecstasy use-related behaviour (e.g. trying out ecstasy, ceasing ecstasy use, getting ecstasy tested, or drinking water during use). The aim of this overview is to guide further quantitative research into ecstasy use, eventually enabling development of effective evidence-based interventions.

## Methods

Relevant literature was identified through the databases PsycINFO and MedLine. These were accessed through the Ovid SilverPlatter WebSpirs interface (version 5.12). At the 21^st ^of August 2008, the query "(("ecstasy" OR "mdma" OR "xtc" OR "methyldioxymethamphetamine" OR "party drug" OR "party drugs" OR "club drug" OR "club drugs" OR "dance drug" OR "dance drugs") IN TI, AB) AND (LA = "English")" was entered, which searched for all English records that contain ecstasy (or a synonym) in their title or abstract. This query yielded 4574 hits (1232 from PsycINFO and 2021 from MedLine). The phrase "NOT ("mouse" OR "mice" OR "rat" OR "rats")" was added, which eliminated 1321 hits. The remaining 3253 entries were downloaded and imported into a reference management program [11], which automatically identified and deleted 741 duplicates (defined as entries with the same title and year of publication). The titles and abstracts of the 2512 remaining records were manually inspected for relevance, and all publications reporting reasons for an ecstasy use-related behaviour were acquired. The acquired publications were examined in more detail, and if upon closer inspection a paper turned out to not report any reasons for ecstasy use or a related behaviour, it was excluded accordingly. In total, 2490 publications were excluded.

Most excluded records described biological studies [e.g. [12,13]], followed by a large number of publications describing prevalence of drug use, sometimes combined with demographic variables [e.g. [14,15]]. A number of studies also investigated consequences, perceived effects, or risks of ecstasy use [e.g. [16,17]]. Unless these were reported in response to a question about reasons, or considered as reasons by the author of the original paper, these were not considered as reasons in the current paper either. Also, studies not reporting original empirical data were excluded [e.g., discussions or reviews, see for example [18,19]]. Finally, studies that did not investigate the target population (i.e. young recreational ecstasy users in western society) were excluded [e.g. [20,21]], as it has been shown that factors influencing behaviour can differ between populations [22-24].

## Results

### Included studies

Details of the included 22 publications [25-46] are provided in Table 1. The included studies examined several behaviours, and given the qualitative or exploratory quantitative nature of these data, this renders presentation of all results challenging. In 2006, Baylen and Rosenberg [47] reported a review with a goal similar to the current goal, and with resulting data that were structured similarly. As the way in which they report their results seems very useful for the current purposes, this approach will roughly be followed. Specifically, we will report the percentages that were reported in each study in a table, grouped by reason category (rows) and behaviour (columns). Two groups of behaviours share a number of reasons, and the results pertaining to these groups of behaviours are therefore presented in the same table. Table 2 contains four "more-use behaviours": behaviours leading to consumption of more ecstasy (starting use, "using ecstasy" in general, using more ecstasy, and not ceasing ecstasy use). Table 3 contains three "less-use behaviours": behaviours leading to consumption of less ecstasy (not starting use, using less ecstasy, or ceasing use). In addition to these seven behaviours, a number of studies addressed reasons for combining ecstasy with other drugs and applying harm reduction strategies [25,28,29,35,36,40,46]. Because of the multitude of different behaviours, these reasons will not be tabulated but rather discussed in the text.

**Table 1:** Authors and publication years of the included studies, and the letter denoting these studies.

**Authors and number in reference list**	**Year**	l*	**Country**	**Time**	**Sampling method**	**Measurement**	**N**	**% ♀**	**Age**
Solowij, Hall & Lee [40]	1992	A	Australia	NR	RDS	Questionnaire	100	39%	27
Fountain, Bartlett, Griffiths, Gossop, Boys & Strang [32]	1999	B	UK	NR	Selected sample with diverse experience with drugs	Interview	100	36%	18
Topp, Hando, Dillon, Roche & Solowij [43]	1999	C	Australia	NR	RDS, advertisement, radio, flyers	Interviews	329	51%	23
Boys, Marsden & Strang [27]	2001	D	UK	August-November 1998	RDS	Questionnaire	364	44%	19
Hansen [35]	2001	E	Australia	July 1998-February 2000	Explicit selection	Participant observation & interviews	31	42%	25
Winstock, Griffiths & Stewart [46]	2001	F	UK	June 1999	Questionnaire in magazine	Questionnaire	1151	40%	24
Dundes [30]	2003	G	US	October 2000	Distribution by students	Questionnaire	719	55%	20
Fendrich, Wislar, Johnson & Hubbell [31]	2003	H	US	June 2001-January 2002	Random selection	Audio Computer self-interview	627	61%	28
Verheyden, Henry & Curran [44]	2003	I	UK	NR	Sampling in bars, private residences, clubs, universities, offices	Questionnaire guided interview	430	45%	24
Verheyden, Maidment & Curran [45]	2003	J	UK	NR	Sampling of ex-users from other study	Questionnaire	47	0%	30
Carlson, Falck, McCaughan & Siegal [28]	2004	K	US	Spring 2001-Winter 2002	Convenience sample, RDS	Focus groups & interviews	30	50%	22
Gourley [34]	2004	L	Australia	NR	Explicit selection	Interviews & observations	12	50%	21
Riley & Hayward [37]	2004	M	UK	February-March 2001	Sampling at dance venues	Questionnaire	124	50%	25
Gamma, Jerome, Liechti & Sumnall [33]	2005	N	US**	NR	Links at websites	Online survey	923	NR	19
Levy, O'Grady, Wish & Arria [36]	2005	O	US	2003	Flyers	Focus groups	30	57%	20
Soellner [39]	2005	P	Germany	1994–1998	Random sample	Computer assisted interviews	2246	NR	NR
Allott & Redman [25]	2006	Q	Australia	June-December 2004	Convenience sample, RDS, advertisement	Questionnaire	116	51%	27
Copeland, Dillon & Gascoigne [29]	2006	R	Australia	NR	NR	Interviews	216	47%	26
Rodgers, Buchanan, Pearson, Parrott, Ling, Hefferman & Scholey [38]	2006	S	US, EUR**	NR	Links on websites	Online questionnaire	209	40%	16–20
Sumnall, Cole & Jerome [42]	2006	T	US, UK, Australia, Eire**	NR	RDS, printed posters, advertisement, key informant access	Questionnaire	268	37%	26
Sterk, Theall & Elison [41]	2007	U	US	NR	Respondent driven sampling	Computer assisted interviews	261	30%	21
Bellis, Hughes, Calafat, Juan, Ramon, Rodriguez, Mendes, Schnitzer & Phillips-Howard [26]	2008	V	Portugal, Spain, Italy, Greece, Slovenia, Czech Republic, Austria, Germany, UK	NR	RDS	Questionnaire	146	49%	21

* = letter used in Tables 2 and 3 to refer to this study, ** = probably primarily these region(s) (internet study), US = United States, UK = United Kingdom, EUR = Europe, RDS = respondent driven sampling (e.g. snowballing), NR = not reported

**Table 2:** Reasons and reported frequencies in each included study for starting ecstasy use, using ecstasy, using more ecstasy, and not ceasing ecstasy use.

**Reason categories (reasons as reported in original papers in parentheses)**	**Starting ecstasy use**	**Using ecstasy**	**Using more ecstasy**	**Not ceasing ecstasy use**
Availability/price/quality of ecstasy (being offered an ecstasy pill, lower cost of ecstasy^E^; ecstasy quality... decreased, increased^F^; I have more money to spend^I^; availability of ecstasy^M^; availability ('was there so I tried it')^O^; friend offered and felt I could not decline^U^)	NN^O^	NN^E^; 27%^U^	NN^E^; 21%, 35%^F^; 7%^I^; NN^M^	
Changing life circumstances (moving in or out of a certain lifestyle) (it is part of my lifestyle^I^)			14%^I^	
Curiosity (out of curiosity, for experimental reasons^A^; curious about good experiences of others, general interest in effects of psychoactive substances^K^; the hype surrounding ecstasy^L^; curiosity^O^)	NN, NN^A^; NN, NN^K^; NN^L^; NN^O^			
Decreased drug effects (e.g. tolerance) or decreased appreciation of drug effects (needing to take more tablets than used to^F^; I need to take more to get the same effects^I^; increased tolerance^K^)			35%^F^; 9%^I^; NN^K^	
Denying or forgetting negative effects (thinking "that won't happen to me" or "well, everybody else is doing ecstasy, and they're not having any problems", upon hearing about negative consequences^K^; unpleasant experiences are forgotten and the excitement of going out and socialising takes over^L^)				NN^K^; NN^L^
Desire to be on the same level as friends (i.e. to be intoxicated in the same way) (to get into the spirit of the party^H^; it makes you sad if you're at a club and you see everybody else is having all this fun and you're not^K^; having a shared experience, desire to be on the same level as friends^L^; social pressure ("you see friends having a great time and you want to join")^O^	NN^K^; NN^O^	70%^H^; NN, NN^L^		
Ease of administration (controlled freedom/sense of control, provides fun, confidence and companionship that users seek without negative consequences associated with other drugs, effects preferred to those of alcohol^E^; using ecstasy is more convenient than using alcohol^L^; ease of use in comparison to other drugs^O^)	NN^O^	NN, NN, NN^E^; NN^L^		
Enhance energy and dancing (help you to... keep going on a night out with friends, stay awake^D^; to stay up longer, to dance/be more active^H^; enable partying all night an makes the fun and excitement of the night last longer^L^; staying awake, enhancing dancing, dance energy^M^; stimulation^P^; dancing^T^)		91%, 72%^D^; 39%, 57%^H^; NN^L^; NN, NN, 60%^M^; NN^P^; 59%^T^		
Enhance mood (to feel good) (for fun^A^; make yourself feel better when down or depressed, help you feel elated or euphoric^D^; enhance mood^L^; hedonistic pleasure, for a laugh, loved up feeling^M^; positive effects on mood, desire to have fun^O^; a desire to feel good^P^; fun^T^)	NN^A^; NN, NN^O^	48%, 78%^D^; NN^L^; NN, 56%, NN^M^; 47%^P^; 42%^T^		
Enhance other substances' effects (improve the effects of other substances, help ease the after effect of other substances^B^)		27%, 8%^B^		
Enhance sex (enhance feelings when having sex^D^; to enjoy sex more^H^; increased sexual please, feeling more emotionally connected to partners during sex^O^; enhance sex^T^; prolong erection, enhance sexual sensations and arousal, unusual/exciting sexual activity^V^)		62%^D^; 22%^H^; NN, NN^O^; 29%^T^; 10%, 23%, 21%^V^		
Enhance social interaction (help you to... enjoy the company of friends, feel more confident or more able to talk to people^D^; affirmation of friendships, ecstasy facilitates particular social activities^E^; I am more open with people, I am more confident^I^; enhancing socialising, for socialising/confidence, to pull/have sex, openness^M^; affiliation, being together with other people^P^; sociable^T^; facilitate sexual encounter^V^)		63%, 42%^D^; NN, NN^E^; NN, 65%, 20%, NN^M^; NN, 71%^P^; 53%^T^; 12%^V^	3%, 2%^I^	
Enhance/change sensory perception (help make something you do less boring, enhance an activity such as listening to music^D^; sensory sensations^E^; to alter perspective^M^; to produce altered states of consciousness, creative, to enjoy music^T^)		36%, 80%^D^; NN^E^; 47%^M^; 70%, 29%, 56%^T^		
Experienced no or unpleasant ecstasy effects (ecstasy experience does not live up to expectations^E^; not feeling any effect of the ingested ecstasy pills^L^; did not feel it the first time^U^)		11%^U^	NN^E^; NN^L^	
Experienced very pleasant effects (ecstasy experience is particularly good^L^; liked what it did for me, thought subsequent experiences would be same/better than first^U^)		93%, 89%^U^	NN^L^	
Fear of health risks (worrying about... dying from ecstasy, risk of brain damage^F^)			1%, 1%^F^	
Feeling safe about ecstasy contents and ecstasy use setting (being certain about what is ingested and that an organisation of knowledgeable volunteers is present^G^)	19%^G^		51%^G^	
Help lose weight (help you to lose weight^D^)		7%^D^		
Help you to concentrate, work, or study (help you to concentrate or to work or study^D^)		3%^D^		
Intoxication, losing inhibitions (just get really stoned or intoxicated, help you to lose inhibitions^D^; loss of inhibitions^E^; just to get high/enjoy oneself^H^; to lose it (being uninhibited)^M^; desire for an altered state of mind ("desire to get screwed up")^O^)	NN^O^	68%, 50%^D^; NN^E^; 91%^H^; 31%^M^		
Noticed mood/affective/cognitive changes in oneself (feeling depressed a few days after use^F^)			1%^F^	
Other's bad experience/death/mood/affective/cognitive changes (knowing someone who has had a bad experience on ecstasy^F^)			1%^F^	
Own bad experience (having a bad experience on ecstasy^F^)			1%^F^;	
Positive effects outweigh negative effects (positive effects seem to outweigh risks; positive effects from use outweigh the negative effects^E^; ecstasy use feels too good despite worries about depression^K^)	NN^E^			NN^E^; NN^K^
Presence of opportunity (raves^T^)		58%^T^		
Recreation/relaxation/stop worrying (recreational purposes^A^; help you to... relax, stop worrying about a problem^D^; a time out from the normal routine and stress of daily life^K^; being at a major dance event, relax or unwind^L^; boredom, to switch off/relax, to escape problems/worries/out of boredom^M^; boredom, desire to escape^O^; relaxation, to party, to have a good time, coping with problems, as a distraction^P^)	NN^A^; NN, NN^O^	30%, 33%^D^; NN^K^; NN, NN^L^; NN, 69%, 32%, 21%^M^; NN, 57%, 62%, 11%, 14%^P^		
Self-medication (enables socially anxious individuals and/or those with low self-esteem and confidence to fit in with others and have a good time, provides temporary relief from depressive symptoms^O^; insecurity^P^; personal 'psychotherapy', group 'psychotherapy'^T^)	NN, NN^O^	6%^P^; 42%, 24%^T^		
Social influence (friends use ecstasy) (most of my friends take it^I^; being with friends who take the drug, desire to continue interacting with an ecstasy-using group of peers^L^; because mates take it, peer-group behaviours^M^; wanted to be accepted by friends^U^)		20%^M^; 8%^U^	6%^I^; NN^L^; NN^M^	NN^L^
Spirituality (spiritual, close to nature^T^)		21%, 23%^T^		

Note: superscripted letters denote studies as listed in Table 1, NN = no numbers (frequency or percentage) reported

**Table 3:** Reasons and reported frequencies in each included study for not starting ecstasy use, using less ecstasy, or ceasing ecstasy use.

**Reason categories (reasons as reported in original papers in parentheses)**	**Not starting ecstasy**	**Using less ecstasy**	Ceasing ecstasy use*
Addiction, fear of becoming dependent (fear of addiction^B^, feeling dependent on ecstasy^C^, addiction/tolerance^O^, addiction^P^)	0%^B^	16%^C^	NN^O^; 36.3%^P^
Availability, price, quality of ecstasy (financial reasons, high price of ecstasy^A^; financial cost^B^; financial difficulties^C^; knowing that a pill does not contain MDMA, monetary factors, quality factors^E^; ecstasy quality... decreased, increased^F^; perceived drop in ecstasy quality, money is a problem^I^; money problems, MDMA quality^J^; availability of ecstasy^M^; money^O^)	NN^A^; 2%^B^;	57%^C^; NN, NN, NN^E^; 34%, 10%^F^; 34%^I^; NN^M^	NN, NN^A ^*; 34%^I^; 1.4, 6.3^J ^*; NN^O^
Changing life circumstances (moving in or out of a certain lifestyle) (having decided not to do drugs anymore^A^; changes in life circumstances^E^; I'm getting older, if I was spending less time at clubs, if I was spending less time at pubs, if I was spending less time at parties^I^; stopped clubbing^J^; growing out of the scene^L^; loss of interest^O^; moving on^S^)		NN^E^; 12%^I^; NN^L^;	NN^A ^*; 30%, 12%, 7%^I^; 5.1^J ^*; NN^O^; 16%^S^
Lack of curiosity (uninterested in the effects, unfamiliarity with the drug and/or its effects^B^)	18%, 2%^B^		
Decreased drug effects (e.g. tolerance) or decreased appreciation of drug effects (e.g. getting bored by effects) (needing to take more tablets than used to^F^; I'm not getting the same rush as I used to get^I^; bored of the drug's effects^M^)		9%^F^; 18%^I^; NN^M^	
Ecstasy is overrated (ecstasy is boring or overrated^A^; not every ecstasy experience is necessarily as good as the last^L^)		NN^L^	25%^A ^*
Experienced no effects or unpleasant effects (experience was unpleasant, found the experience boring^A^; not enjoying drug^J^; intensity of first experience was overwhelming and not worth the trouble of continuing to use^K^; ecstasy did nothing to me^P^)	25%, 41%^A^		5.6^J ^*; NN^K^; 44%^P^
Fear of ecstasy's effects (fear of the effects^B^)	43%^B^		
Lack of opportunity (having had no opportunity to take ecstasy^A^; lack of opportunity^B^)	NN^A^; 10%^B^		
Legal consequences (external circumstances (legal)^E^; getting a criminal record^I^; criminal record^J^; fear of legal consequences^O^)			7%^E^; 10%^I^; 1.2^J ^*; NN^O^
Minimising ecstasy comedown (avoiding the ecstasy comedown^Q^)		56%^Q^	
Minimising health risks or fear of health risks (wariness regarding the effects of ecstasy, health reasons^A^; fear of physical harm, fear of psychological harm^B^; physical health effects, psychological problems^C^; potential health risks, minimise the potential for negative or adverse outcomes^E^; worrying about... dying from ecstasy use, risk of brain damage^F^; fears about... long-term effects on mental health, long-term effects on physical health, short-term effects on mental health, short-term effects on physical health^I^; long-term mental health, short-term mental health^J^; avoid potential risks^K^; health concerns^O^; fear of damage to health^P^; avoiding ecstasy-related negative side-effects, avoiding brain damage or neurotoxicity^Q^; negative effects^S^)	NN^A^; 33%, 0%^B^	45%, 39%^C^; NN, NN^E^; 15%, 25%^F^; NN, NN^K^; 71%, 58%^Q^	NN^A ^*; 67%, 46%, 17%, 13%^I^; 5.8, 4.5^J ^*; NN^O^; 62%^P^; 14%^S^
Noticed mood/affective/cognitive changes in oneself (external circumstances (medical)^E^; feeling depressed a few days after use^F^; finding it was doing my head in, it takes it out of you physically, I get depressed, I have some memory loss, it takes longer to come down, I have not been feeling healthy, it makes me less tolerant to others^I^; depressed, paranoia, anxiety, memory, concentration, physical health worries, impulsive behaviour, sleeping worries, angry, eating worries^J^; depression^M^)		27^F^; 30%, 17%, 13%, 13%, 12%, 6%^I^; NN^M^	7%^E^; 50%^I^; 5.6, 5.4, 5.3, 5.1, 4.9, 4.3, 3.3, 3.1, 3.0, 2.9^J ^*
Observation of others using ecstasy (seen the effect on others^B^; observation of others using ecstasy^O^)	16%^B^		NN^O^
Other's bad experience/mood/affective/cognitive changes/death (knowing someone who had a bad experience on ecstasy^F^; seeing someone have a bad experience on MDMA, knowing someone who... died as a result of taking MDMA, became mentally ill, became physically ill^I^; other's bad experience, other mentally ill^J^; other's bad experiences^M^)		11%^F^; NN^M^	31%, 19%, 17%, 14%^I^; 2.9, 2.2^J ^*
Own bad experience (having a bad experience on ecstasy^F^; personally having a bad experience on MDMA^I^; bad experience^J^; own bad experience^M^; problems caused by ecstasy^N^; negative personal experiences^O^)		22%^F^; NN^M^	25%^I^; 3.4^J ^*; 60%^N^; NN^O^
Responsibilities (interference with or increase/decrease in) or relationship problems (occupational problems, to improve quality of life, relationship problems^C^; social factors^E^; it places strains on my job/studies, I have more responsibilities, if I thought it... was negatively influencing my work/study, might affect my job^I^; work affected^J^; fear of reduced efficiency^P^)		28%, 17%^C^; NN^E^; 19.6%, 11.3%^I^	NN^A ^*; 37%^C^; 18%, 16%^I^; 4.7^J ^*; 75%^P^
Social influence (friends quit using ecstasy) (peer influence^B^; if friends were giving up, most of my friends have given it up^I^; friends quit^J^; peer-group behaviours, being with people who don't use (many) drugs^M^)	7%^B^	9%^I^; NN, NN^M^	22%^I^; 1.8^J ^*
Social influence from relatives (pressure from relatives, relatives finding out I was taking MDMA^I^; relatives finding out, relatives' pressure^J^)			2%, 2%^I^; 2.0, 1.7^J ^*

Note: superscripted letters denote studies as listed in Table 1, * Study A reports reasons to not use ecstasy for 1–3 time users, and study J reports scores to indicate relevance of each reason on a 10-point scale, reported by ex-users, NN = no numbers (frequency or percentage) reported

The authors have clustered the reasons in Tables 2 and 3, but exclusively to ease presentation and discussion, as the qualitative nature of this review prohibits quantitative integration of the results. These categories were established by first entering all reasons into an online database [where they are available to the interested reader; see [48]]. Then, the first author clustered those reasons that appeared similar, eventually reaching a list of relatively distinct categories. The clustering does not suggest that the grouped reasons are psychologically similar, but rather only serves to ease presentation and discussion of the results. Therefore, the original descriptions for each reason are listed in the first column of every table. In addition, interested readers can consult the original (unclustered) lists of reasons, which have been made publicly available [48]. The descriptions are provided in the same order as the corresponding reporting frequency (if available). When several reasons within one category were extracted from one study, the descriptions and reporting frequencies are separated by commas.

### More-use behaviours

A number of patterns emerge when all studies into starting use, "using ecstasy" in general, using more ecstasy, and not ceasing ecstasy use are combined (see Table 2). First, like studies in the meta-analysis, most currently reviewed studies focused on the behaviour 'using ecstasy'. However, there is still a lot of data on other behaviours, such as starting to use ecstasy, using more ecstasy, and not ceasing ecstasy use. The reason categories in which the reasons for these behaviours fall have been summarised in Table 4. In this table, a tentative attempt has been made to indicate each reason category's relevance, based on the frequency with which the reasons in a category were endorsed by participants. When at least one reason in a reason category was endorsed by more than half of the participants, a reason category was considered very relevant (indicated in the table by '+'); when reasons in a reason category were reported by less than half, but more than one in ten participants, a reason category was considered moderately relevant ('±'); and when reasons in a reason category were reported by one in ten participants or less, the category was considered minimally relevant ('-'). When no frequency information was available (i.e. with interview studies where only quotes were provided), the symbol 'N' is used, and in the one case where the only study suggested that a reason was irrelevant, the symbol '✘' is used.

**Table 4:** Overview of the reason categories in which one or several reasons were reported for each behaviour

**Reason categories**	**Starting ecstasy use**	**Using ecstasy**	**Using more ecstasy**	**Not ceasing ecstasy use**	**Not starting ecstasy**	**Using less ecstasy**	**Ceasing ecstasy use**
Addiction, fear of becoming dependent					✘	±	±
Availability/price/quality of ecstasy	N	±	±		-	+	±
Changing life circumstances (moving in or out of a certain lifestyle)			±			±	±
Curiosity (or lack of curiosity)	N				±		
Decreased drug effects or decreased appreciation of drug effects			±			±	
Denying or forgetting negative effects				N			
Desire to be on the same level as friends (i.e. to be similarly intoxicated)	N	+					
Ecstasy is overrated						N	±
Ease of administration	N	N					
Enhance energy and dancing		+					
Enhance mood (to feel good)	N	+					
Enhance other substances' effects		±					
Enhance sex		+					
Enhance social interaction		+	-				
Enhance/change sensory perception		+					
Experienced no or unpleasant ecstasy effects		±	N		±		±
Experienced very pleasant effects		+	N				
Fear of ecstasy's effects					±		
Feeling safe about ecstasy contents and ecstasy use setting	N		+				
Help lose weight		-					
Help you to concentrate, work, or study		-					
Intoxication, losing inhibitions	N	+					
Legal consequences							±
Minimising ecstasy comedown						+	
Minimising health risks or fear of health risks					±	+	+
Noticed mood/affective/cognitive changes in oneself						±	+
Observation of others using ecstasy					±		N
Other's bad experience/mood/affective/cognitive changes/death						±	±
Own bad experience						±	+
Positive effects outweigh negative effects	N			N			
Presence or lack of opportunity		+			±		
Recreation/relaxation/stop worrying	N	+					
Responsibilities or relationship problems						±	+
Self-medication		±					
Social influence (friends use ecstasy or quit using ecstasy)		±	-	N	-	-	±
Social influence from relatives							-
Spirituality		+					

Note: + denotes highly relevant categories; ± denotes moderately relevant categories; -denotes minimally relevant categories; N denotes that no relevance information was available; ✘ denotes irrelevant reasons.

Three reasons from Table 2, specifically fear of health risks, noticing mood/affective/cognitive changes in oneself, and one's own or another's bad experience, were each reported as reasons for using more ecstasy by 1% of the participants of study F [46]. The current authors assumed that this reflects measurement error, and upon being contacted, the original authors confirmed that they share this assumption. These reasons have therefore been omitted from Table 4.

When this information is combined for all more-use behaviours, it becomes clear that although some reason categories are equally relevant for all behaviours, there are also differences. Understandably, curiosity only seems relevant for starting ecstasy use; denial of negative effects only seems relevant for not ceasing use; and tolerance is only relevant for using more ecstasy. However, other differences are less intuitive. For example, social influence, and ecstasy's ability to provide energy and enhance social interaction and sensory perception, do not seem to play a big role in starting to use ecstasy.

### Less-use behaviours

When looking at behaviours that health promoters would generally construe as the desirable behaviours, it is clear that most research focussed on using less ecstasy and ceasing ecstasy use (see Table 3). Although the reasons for using less ecstasy and ceasing ecstasy use were quite similar, different reasons were reported for not starting ecstasy (see Table 4). For example, the cost of ecstasy does not deter potential users, but it does cause users to use less or even cease use, and other people's bad experiences can be a reason to use less ecstasy or cease altogether, but was not reported as a deterrent by non-users. Fearing or minimising health risks was reported for all three behaviours, although markedly less frequently as a deterrent to not start using ecstasy. When comparing these reasons with the 'more-use behaviours', it became clear that there was very little overlap. It seems that people have different reasons for starting ecstasy use and for not starting ecstasy use, and yet different reasons for using less ecstasy and for ceasing ecstasy use, and yet again for using ecstasy.

### Combining drugs and applying harm reduction strategies

In total, seven studies reported reasons to combine ecstasy with other drugs, to apply harm reduction strategies, or to refrain from these behaviours. Five studies reported reasons to combine ecstasy with other drugs, and all reasons fell in one of two categories [29,35,36,40,46]: to enhance the ecstasy experience, or to minimize the comedown. To enhance the ecstasy experience, ecstasy was combined with ADHD medication, amphetamine, benzodiazepines, ketamine, LSD, marijuana, and Viagra (studies A [40], E [35], O [36] and R [29]). To minimize the comedown, ecstasy was combined with alcohol, antihistamine, benzodiazepines, cocaine, heroin, ketamine, marijuana, oxycodone-containing analgesics, rohypnol and valium (studies A [40], E [35], F [46], O [36] and R [29]). Interestingly, studies also reported that people *refrained *from combining with other drugs to maximize the ecstasy experience (studies A [40] and K [28]). Other reasons to refrain from combining were to minimize health risks (studies E [35] and K [28]) and after having heard about people dying from ecstasy use (study K [28]). To minimize health risks, participants also pre- or postloaded with vitamins, 5-Hydroxytryptophan (5-HTP), or selective serotonin re-uptake inhibitors (SSRIs; studies O [36], Q [25] and R [29]). Preloading was also reported to enhance the ecstasy experience (studies Q [25] and R [29]), and postloading to minimize the comedown (studies Q [25] and R [29]), and one study reported that participants drank water during use to minimize the comedown (study Q [25]).

Most other harm reduction strategies were applied to minimize the potential for negative or adverse outcomes or health risks, namely drinking water and chilling out during ecstasy use (both from study Q [25]; chilling out means taking breaks from dancing), purchasing fewer ecstasy pills per occasion and limiting one's supply, only using when in a positive mood and with friends, and the more altruistic behaviours of guiding initiates and monitoring others (all from study E [35]). Then, a number of behaviours served to deal with the uncertain contents of ecstasy pills: using only after someone else had tried the ecstasy (study E [35]), obtaining pills from a reliable source (studies K [28] and O [36]), and purchasing pills in bulk (study E [35]). However, one study also reported that participants could avoid getting their ecstasy tested because they considered the uncertainty (as to the pill contents) 'part of the process' (study E [35]). Finally, one study reported a user who liked to drive under the influence of ecstasy because he enjoyed the experience (study E [35]).

## Discussion

The papers included in this review contain valuable information. Compared to the synthesis of quantitative literature [8], the studies included here have indeed addressed more behaviours and more potential determinants. Though a minority of reasons reported here has already been quantitatively studied, those quantitative studies have only examined their relevance for the behaviour 'using ecstasy', and the results show that reasons for different behaviours (e.g. 'using ecstasy' and starting or ceasing ecstasy use) differ. This means that an intervention targeting the important determinants for 'using ecstasy' may be unable to effectively influence other behaviours (such as starting or ceasing ecstasy use). This also means that development of evidence-based interventions addressing these other behaviours first requires studies that map the determinant configurations for those specific behaviours.

Unfortunately, this review cannot inform intervention development, because this review only provides an overview of how frequently a reason was reported, and comparison of the frequency with which reasons were reported with the effect sizes found in the meta-analysis for the behaviour 'using ecstasy' showed that frequently reported reasons can correspond to beliefs that were not associated to frequency of use (i.e. beliefs held equally strongly by users and abstainers or by heavy users and light users). For example, in this review, using to 'enhance energy and dancing' was mentioned as a reason for using ecstasy by between 39% and 91%, yet in the meta-analysis [8], the belief that ecstasy helps to stay awake was associated to ecstasy use with a trivial effect size (i.e. Cohen's d < .2 [49]). A second limitation of this review is the fact that with two exceptions [26,39] all included studies have been performed in the US, the UK and Australia. It remains to be seen whether these conclusions apply to other countries such as the Netherlands. Third, following from the qualitative methodology, no conclusions can be drawn except that reasons for related but different behaviours differ; nothing can be said about the degree to which they differ. This conclusion does, however, imply that determinant configurations (i.e. relative relevance of each of the determinants of a behaviour) of related but different behaviours differ as well.

Thus, there is a need to find out whether and to what degree determinant configurations for ecstasy use-related behaviours differ, ideally by comparing one or more behaviours (e.g. trying out ecstasy, using ecstasy and ceasing use) in one study. If these determinant structures do indeed differ, interventions should target different determinants depending on the specific behaviour that is targeted. In addition, future studies should measure the beliefs underlying the reasons for each behaviour. Ideally, for each behaviour, beliefs potentially underlying all reasons that have been studied (i.e. that have been marked in Table 4) are quantitatively examined. That way, over time, a clear picture will emerge as to the relative relevance of each of these reasons.

Just after the current review was completed, two new manuscripts were published that also addressed reasons to refrain from trying out ecstasy [50,51]. Vervaeke, Benschop and Korf conducted a factor analysis and found support for three factors: fear of the effects, rationality, and lack of opportunity [50]. Rosenberg, Baylen, Murray, Phillips, Tisak, Versland and Pristas used a different method and distinguished eight factors: harm to thinking, school, work, or athletic performance; ecstasy use is contrary to values/self-image; fear of failing a drug-test; fear of effects on body; difficulty with acquiring ecstasy; fear of dangerous outcomes; no enjoyment expected from ecstasy; and fear of loss of control. Most reasons underlying these factors reflect reasons from the earlier studies that were included in this review, but additional reasons to refrain from starting ecstasy use are also reported: uncertainty about pill contents, medical reasons, no access to ecstasy, already using another substance, and not using on principle [in [50]], and against religion, fear of damage to reputation, want to be a role model, don't know where to get it, and fear of losing control [in [51]]. Especially interesting are the different factor structures revealed by these two studies. This may be attributed to their different methodologies of constructing the factors, or to the different locales (Dutch versus American).

## Conclusion

The results of this review provide a clear agenda for the research needed to develop evidence-based interventions addressing ecstasy use. Worth noting in this respect is that many studies reported overlapping reasons, both within and between studies. For example, it is unclear whether, and if so, to what degree, the reasons "help enjoy the company of friends", "enhance socialising", and "being together with other people" reflect similar determinants. Ideally, a number of largely orthogonal beliefs can be identified [by studies such as [50] and [51]], the relevance of each of which can then be established for each behaviour. As multiple theoretical frameworks seem to apply to ecstasy use [8], it seems advisable for future studies to include variables specified by different theories so that it can be determined whether and how the relevant beliefs underlie these variables.

Finally, the combination of this study and the meta-analysis [8] has important implications. First, by virtue of their strict quantitative approach, meta-analyses provide only a very narrow view into the literature, excluding many studies that may provide valuable pointers for future research. By considering these excluded studies, qualitative reviews remain very valuable tools in synthesising the state of the literature. Second, conclusions from such qualitative reviews need to be quantitatively verified. As was also the case in the current review, results from qualitative research may not be corroborated by quantitative data. Thus, a balanced synthesis of the state of the art requires both meta-analytical and qualitative reviews.

## Competing interests

The authors declare that they have no competing interests.

## Authors' contributions

GJYP conceived of and conducted the study and the analyses and drafted the manuscript. GK contributed to the conceiving of the study and to the interpretation of the data and helped to draft the manuscript. Both authors read and approved the final manuscript.

## Pre-publication history

The pre-publication history for this paper can be accessed here:


